# Circulating Blood miR-155 and miR-21 Promote the Development of Acute Pancreatitis and Can Be Used to Assess the Risk Stratification of Pancreatitis

**DOI:** 10.1155/2021/2064162

**Published:** 2021-12-14

**Authors:** Lan Hu, Dongdong Han, Diao Yu, Dongji Ao, Zhengyi Yang

**Affiliations:** ^1^Department of Gastroenterology, Bijie First People's Hospital, Bijie 551700, Guizhou Province, China; ^2^The Second People's Hospital of Dongying City, Dongying 257300, Shandong, China; ^3^Department of Laboratory Medicine, Bijie First People's Hospital, Bijie 551700, Guizhou Province, China

## Abstract

To explore the role of circulating blood miR-155 and miR-21 in promoting acute pancreatitis (AP) and evaluating the risk stratification of pancreatitis. In this experiment, 70 patients with AP treated in our hospital from October 2019 to December 2020 were included in the research group (RG), and the blood of 52 healthy cases was collected and they were included in the control group (CG). The expression of miR-155 and miR-21 in circulating blood was observed in the two groups. The diagnostic efficacy of miR-155 and miR-21 in AP was observed. The risk factors of patients with AP were observed. The expression of serum gastrointestinal hormones was observed in the two groups. The GAS and VIP in RG were higher than those in CG, while MTL and CCK were lower than those in CG. Moreover, the detection level of mild, moderate, severe, and critical patients was also significantly different (*P* < 0.05). The expression of miR-155 and miR-21 in circulating blood of RG was significantly lower than that of CG (*P* < 0.05), and the area under the miR-155 curve was 0.775 and the area under the miR-21 curve was 0.832. Alcoholism, GAS, VIP, MTL, CCK, miR-155, and miR-21 were the risk factors of patients. miR-155 and miR-21 show low expression in the serum of patients. The lower the expression, the more serious the disease. They are closely related to the development of AP. miR-155 and miR-21 have good diagnostic efficacy by ROC analysis, and they are expected to become effective indicators for the diagnosis and treatment of AP in the future.

## 1. Introduction

Pancreatitis is a major cause of gastrointestinal disease-related diseases, which is related to high morbidity, mortality, and social and economic burden [1]. The incidence of AP is different all over the world [2]. According to WHO definition [3], the high-incidence areas (i.e., areas with an annual incidence exceeding 34 cases per 100,000 people) are North America and Western Pacific. As a whole, Europe is a low-incidence area (there are 29 cases per 100,000 ordinary people every year). It has been revealed that the incidence of AP varies throughout the European continent, and Northern Europe and Eastern Europe are the most affected [4]. Nevertheless, due to the lack of excellent research from Eastern and Southern Europe, it is difficult to compare the morbidity of AP in Europe in a powerful way [5]. In view of this situation, we urgently need to find a new potential target for treatment and diagnosis and further clarify the development of pancreatitis to improve the current situation.

With the deepening of research, scholars at home and abroad began to focus on gene research in recent years. miRNA (microRNA) is a kind of small noncoding RNA, which can be applied as endogenous RNA interference to adjust the targeted genes and affect the regulation of various physiology and pathologic functions [6]. Bioinformatics data reveal that a single miRNA can bind to hundreds of target mRNA, thus playing a crucial role in various biological processes. At present, it has been proved to be closely related to the development and progression of various human tumor diseases [7, 8]. miRNA is a protein regulator, which plays an important role in various cell functions [9]. miR-155 has a series of known biological functions, including inducing the activation of Toll-like receptors (TLR) and regulating TLR signaling transduction in monocytes/macrophages, thus promoting inflammatory cell reactions and triggering systemic inflammatory reactions [10, 11]. Research studies have revealed that [12] miR-21 is also closely bound up with the development and progression of pancreatitis. Therefore, we will verify our conjecture through experimental analysis, so as to provide references and guidance for clinical diacrisis and therapy of pancreatitis in the future. Our study aims to explore the role of circulating blood miR-155 and miR-21 in promoting acute pancreatitis (AP) and evaluating the risk stratification of pancreatitis.

## 2. Materials and Methods

### 2.1. Baseline Data

From October 2019 to December 2020, 70 cases with AP admitted to our hospital were included in the RG and the blood of 52 healthy cases was collected and they were included in the CG in this experiment. In RG, there were 41 men and 29 women with a mean age of 46.6 ± 4.3 years. Disease degree: mild symptoms, there were 17 mild cases, 20 moderate cases, 18 severe cases, and 15 critical cases. In CG, there were 28 men and 24 women with a mean age of 46.2 ± 4.7 years. The collection of clinical data and this test were conducted and ratified by the Medical Ethics Committee of our hospital.

### 2.2. Inclusive and Exclusive Criteria

Inclusive criteria included the following: patients who met the comprehensive diagnosis standard for AP issued by the Chinese Association of Integrated Traditional Chinese and Western Medicine [13]; patients who did not take drugs that affected the test results; patients who cooperated with medical workers to carry out research; patients whose age was 30∼60 years and they had full case materials; patients who were disposed to cooperate with the working schedule of medical workers in our hospital; patients or their immediate dependents who affixed the informed consent form.

Exclusive criteria were as follows: death during therapy, damage to important organs, complicated with other cardio-cerebrovascular diseases, deformity in body, pregnancy, complicated with other autoimmunity diseases, complicated with other chronic illnesses, patients who moved to other hospitals, contraindication of operation, mental disorders, language disturbance, and diseases affecting the findings of this research.

### 2.3. Main Reagents

The gastrin (GAS), vasoactive intestinal peptide (VIP), serum motilin (MTL), and cholecystokinin (CCK), Trizol agent and miRNA reverse transcriptase kit were all purchased from Co., Ltd. TRIzol agent and miRNA reverse transcriptase kit were both from Invitrogen Company. The EasyPure miRNA kit was from Beijing TransGen Biotech Company, China (ER 601-01). Transscript Green miRNA Two-Step qRT-PCR SuperMix was from Beijing TransGen Biotech Company, China (AQ202-01). KH19A desktop high-speed and high-performance centrifuge was from KAIDA Company. The low-temperature refrigerator (−80°C) was from ThermoFisher Scientific Company. The primer sequence of miR-152 was devised and compounded by Sangon Biotech (Shanghai) Co., Ltd. (Table 1).

### 2.4. Collection of Blood Samples

In the early morning, 5 ml of fasting peripheral vein blood was collected from the two groups. Among them, 2 mL of blood samples was stored at 4°C for 30 minutes and centrifuged for 10 minutes (3000 rpm/m). Then, the supernatant fluid was obtained and conserved in a refrigerator at −80°C. In addition, 3 mL of blood samples was tested for miR-155 and miR-21, all of which were processed by the qRT-PCR amplification method.

### 2.5. qRT-PCR Detection and ELISA Detection

The blood samples stored at −80°C were taken out, and the total RNA of tissues was extracted by the TRIzol kit. The purity, concentration, and integrality of the obtained general RNA were tested via ultraviolet spectrophotometry and agarose gel electrophoresis. TransScript Green miRNA Two-Step qRT-PCR SuperMix (AQ202-01, Beijing TransGen Biotech Company, China) was applied for a reverse transcript of the extracted general RNA. The test was conducted according to the kit instructions, and the cDNA was collected for the PCR amplified experiment. The qPCR amplified system was as follows: cDNA (1 *μ*L), upstream and downstream primers (each 0.4 *μ*L), 2 × TransTaq® Tip Green qPCR SuperMix (10 *μ*L), and Passive Reference Dye (50X) (0.4 *μ*L). In the end, ddH_2_O was added to complete to 20 *μ*L. The qPCR-amplified procedures were initial denaturation at 94°C for 30 s, degeneration at 94°C for 5 s, and annealing and extending at 60°C for 30 s, with 40 cycles. Three duplicate holes were established for each specimen, and the test was conducted 3 times in total. In this research, U6 was applied as an internal parameter and 2^−△ct^ was applied to analyze this data. GAS, VIP, MTL, and CCK were obtained in strict accordance with ELISA kit specifications.

### 2.6. Outcome Measures

The main outcome measures were as follows: the miR-155 and miR-21 in circulating blood were observed in the two groups. The diagnostic efficacy of miR-155 and miR-21 in AP was observed. The risk factors of patients with AP were observed.

The secondary outcome measures were as follows: the expression of serum gastrointestinal hormones was observed in the two groups.

### 2.7. Statistical Analysis

In this research, SPSS20.0 was used to statistically analyze the data. GraphPad 7 was applied to plot the requisite pictures. The K-S test was applied to analyze the distribution of dose data, in which normal distribution data were represented via mean number ± standard error (mean ± SD). The independent-samples *t*-test was applied for comparison between groups. The paired *t*-test was applied for comparison within groups. The enumeration data were represented as a percentage. Chi-square tests were applied, denoted by *χ*^2^. ROC was applied to plot the diagnosis efficacy of miR-155 and miR-21 in AP. The single-factor and multifactor logistic regression were applied to analyze the risk factors of patients. There were statistical differences with *P* < 0.05.

## 3. Results

### 3.1. Clinical Materials

There was no obvious difference in clinical data such as age, gender, BMI, smoking history, drinking history, place of residence, exercise habit, and marital status between RG and CG, which proved comparability (*P* > 0.05) (Table 2).

### 3.2. Observing the Expression of Serum Gastrointestinal Hormones in the Two Groups

The GAS and VIP in RG were higher than those in CG, while MTL and CCK were lower than those in CG. Moreover, the detection level of mild, moderate, severe, and critical patients was also obviously different (*P* < 0.05) (Table 3, Figure 1).

### 3.3. Observing the miR-155 and miR-21 in Circulating Blood between the Two Groups

Through qRT-PCR detection, the miR-155 and miR-21 in circulating blood of RG were 0.53 ± 0.46 and 0.81 ± 0.21, while those of CG were 2.86 ± 0.46 and 2.33 ± 0.57. The RG was obviously lower than the CG (*P* < 0.05) (Figure 2).

### 3.4. Observing the Diagnostic Efficacy of miR-155 and miR-21 in AP

According to the expressions of miR-155 and miR-21, ROC was plotted. The findings revealed that the area under the miR-155 curve was 0.775 (*P* < 0.05) and the area under the miR-21 curve was 0.832 (*P* < 0.05) (Table 4, Figure 3).

### 3.5. Univariate Logistic Regression Analysis

According to the degree of illness, the patients were divided into 37 cases with mild or moderate disease and 33 cases with severe and critical illness. Univariate analysis was carried out according to the clinical data in the mild and moderate degree group and severe and critical group. The results revealed that there were no differences in age and gender (*P* > 0.05), but there were differences in alcoholism, GAS, VIP, MTL, CCK, miR-155, and miR-21 (*P* < 0.05) (Table 5).

### 3.6. Multivariate Logistic Regression Analysis

The differential indicators in single factors (alcoholism, GAS, VIP, MTL, CCK, miR-155, and miR-21) were included and assigned (Table 6). Multivariate logistic regression analysis was subsequently performed, and the results were as follows: alcoholism (OR: 3.521, 95% CI: 1.061∼3.183), GAS (OR: 5.020, 95% CI: 0.218∼0.675), VIP (OR: 3.227, 95% CI: 1.072∼2.901), MTL (OR: 4.019, 95% CI: 1.467∼4.218), CCK (OR: 4.629, 95% CI: 1.353∼5.727), miR-155 (OR: 6.786, 95% CI: 8.824∼19.856), and miR-21 (OR: 2.664, 95% CI: 1.347∼8.783). Alcoholism, GAS, VIP, MTL, CCK, miR-155, and miR-21 were the risk factors of patients (Table 7).

## 4. Discussion

AP is an inflammation-induced disease of the pancreas, and the most general cause is gallstones or excessive use of alcohol. AP can range from slight self-limiting diseases requiring only supportive measures to serious diseases with life-threatening complications [14]. Severe illness accounts for about 20–30% of patients, which is a life-threatening disease with a mortality rate of about 15%. The most commonly used taxonomy system of AP is the Atlanta classification and definition revised in 2012 based on international consensus. It has been identified into two stages (early and late) by this classification. The order of severity is divided into mild, moderate, severe, and critical. Mild patients (interstitial edematous pancreatitis) have no organ failure and local or systemic complications, and the disease usually goes away within the first week. If there is transient (less than 48 hours) organ failure, local complications, or deterioration of the disease, it is classified as moderate. Patients with persistent (over 48 hours) organ failure have severe disease forms [15]. Effective biological indicators for diagnosis and treatment of AP are a major research focus in clinics at present.

In this study, miR-155 and miR-21 in patients' serum were tested and the results showed that the miR-155 and miR-21 of patients in RG were lower than those in CG, which revealed that miR-155 and miR-21 were closely related to the development and progression of AP. miR-155, a multifunctional miRNA with inflammatory-related functions, is adjusted by different inflammation media. Bacterial lipopolysaccharide (LPS) and inflammation media, including IFN-*β* and TNF-*α*, can induce miR-155 in human monocyte cell strain. Especially, because it participates in the molecular changes of key targets and signal pathways, the imbalance of miR-155 has been closely related to *Helicobacter pylori*-related gastropathy, inflammatory intestinal disease, and colorectal carcinoma [16–18]. Studies [12, 19, 20] have shown that AP induced by protein in wild-type (WT) mice receiving miR-21 gene knockout (KO) bone marrow is semblable to WT mice transplanted with WT bone marrow, which excludes the possibility of inflammatory invasion. Macrophages or other leukocytes play an important part in the phenotype of less-severe AP in miR-21 KO mice. Therefore, we further mapped ROC. The findings revealed that when the cutoff value was 0.780, the sensitivity and specificity of miR-155 were 67.31% and 78.57%. When the cutoff value was 0.931, the sensitivity and specificity of miR-21 were 86.42% and 71.43%, respectively. They have high diagnostic efficiency, suggesting that miR-155 and miR-21 are expected to be effective targets in diagnosing AP in the future. The expression of serum gastrointestinal hormones was observed in both groups. The findings revealed that GAS and VIP in RG were higher than those in CG, while MTL and CCK were lower than those in CG. There were also significant differences in the detection level of mild, moderate, severe, and critical patients, which indicated that the higher the expression of GAS and VIP, the more serious the patient's condition, while MTL and CCK were opposite. Studies have shown that [21] the age-standardized mortality rate of pancreatitis in China has not changed since 1990. For pancreatitis, alcoholism, obesity, diabetes, and hypertriglyceridemia are some of the risk factors [22], and East-Asian populations are appropriately aware of the risk factors for AP such as regulated metabolism and lifestyle, so it may be different from the western population because of the different relationships between obesity and insulin resistance [23]. At last, we conducted logistic regression analysis and concluded that alcoholism, GAS, VIP, MTL, CCK, miR-155, and miR-21 were the risk factors of patients with AP.

## 5. Conclusion

We have preliminarily revealed the clinical significance of miR-155 and miR-21 through the above research, but there are still some limitations in our study. Firstly, we did not conduct basic cell experiments in this study. Secondly, we did not conduct targeted drug therapy, so we hope to supplement our research results by conducting basic cell experiments and targeted drug therapy in future studies.

In summary, miR-155 and miR-21 show low expression in AP, suggesting that miR-155 and miR-21 are involved in the occurrence and development of AP. Therefore, they are expected to be effective indicators to diagnose and treat AP and to judge the prognosis of patients in the future.

## Figures and Tables

**Figure 1:** Expression level of serum gastrointestinal hormones. (a) Expression level of GAS. (b) Expression level of VIP. (c) Expression level of MTL. (d) Expression level of CCK. Note: the symbol ^*∗*^ indicates that there is a difference between the two groups (*P* < 0.05).

**Figure 2:** Expression of circulating blood miR-155 and miR-21 in the two groups. (a) The expression of miR-155 in RG was significantly lower than that in CG. (b) The expression of miR-21 in RG was significantly lower than that in CG. Note: the symbol ^*∗*^ indicates that there is a difference between the two groups (*P* < 0.05).

**Figure 3:** Diagnostic efficacy of miR-155 and miR-21 in AP. (a) When the cutoff value was 0.780, the sensitivity and specificity of miR-155 were 67.31% and 78.57%, respectively. (b) When the cutoff value was 0.931, the sensitivity and specificity of miR-21 were 86.42% and 71.43%, respectively.

**Table 1:** Primer sequence.

	Upstream sequence	Downstream sequence
U6	5'-ATTGGAACGATACAGAGAAGATT-3'	5'-GGAACGCTTCACGAATTTG-3'
miR-155	5'-GTCCGCTGGCAGTGTCTTAGCTGGTTGT-3'′	5'-GTGCGTGTCGTGGAGTC-3'
miR-21	5'-AACGCTTCACGAATTTGCGT-3'	5'-TGGTGTCGTGGAGTCG-3'

**Table 2:** Basic clinical data (*n* (%)).

	RG (*n* = 70)	CG (*n* = 52)	*χ* ^2^ or *t*	*P*
Age/years	46.6 ± 4.3	46.2 ± 4.7	0.488	0.626
BMI	22.26 ± 0.37	22.21 ± 0.25	0.842	0.402

Gender			0.271	0.603
Male	41 (58.57)	28 (53.85)		
Female	29 (41.43)	24 (46.15)		

Smoking history			0.400	0.527
Yes	37 (61.67)	29 (55.77)		
No	23 (38.33)	23 (44.23)		

Drinking history			0.915	0.339
Yes	33 (47.14)	20 (38.46)		
No	37 (52.86)	32 (61.54)		

Exercise habit			1.111	0.292
Yes	35 (50.00)	31 (59.62)		
No	35 (50.00)	21 (40.38)		

Marital status			0.109	0.742
Married	68 (97.14)	51 (98.08)		
Unmarried	2 (2.86)	1 (1.92)		

Place of residence			0.070	0.791
City	36 (51.43)	28 (53.85)		
Rural	34 (48.57)	24 (46.15)		

**Table 3:** Comparison of serum gastrointestinal hormones between the two groups.

Groups	Cases	GAS (*μ*mol/L)	VIP (*μ*mol/L)	MTL (pg/ml)	CCK (pg/ml)
CG	52	94.24 ± 11.31^a^	2.80 ± 0.34^a^	340.23 ± 26.76^a^	196.25 ± 17.80^a^
Mild	17	102.46 ± 12.63	3.07 ± 0.47	332.15 ± 25.86	188.37 ± 16.35
Moderate	20	127.84 ± 13.79	5.25 ± 0.64	281.27 ± 22.74	160.26 ± 15.19
Severe	18	157.87 ± 16.10	7.42 ± 0.95	186.96 ± 19.86	122.73 ± 13.24
Critical	15	182.94 ± 19.33	9.97 ± 1.17	138.98 ± 15.20	96.64 ± 10.27

Note: compared with the degree of illness, ^*a*^*P* < 0.05; pairwise comparison of disease severity, all *P* < 0.05.

**Table 4:** ROC curve.

	miR-155	miR-21
AUC	0.775	0.832
Std. error	0.046	0.037
95% CI	0.685∼0.865	0.760∼0.904
P	0.001	0.001
Cutoff	0.780	0.931
Sensitivity (%)	67.31	86.42
Specificity (%)	78.57	71.43

**Table 5:** Univariate analysis (*n* (%)).

Clinicopathological features	Mild and moderate (*n* = 37)	Severe and critical (*n* = 33)	*χ* ^2^ or t	*P*
Age/years			0.368	0.607
<30	12(32.43)	13(39.39)		
≥30	25(67.57)	20(60.61)		

Gender			1.496	0.221
Male	23(62.16)	25(75.76)		
Female	14(37.84)	8(24.24)		

Alcoholism			18.500	0.001
Yes	31(83.78)	11(33.33)		
No	6(16.22)	22(66.67)		

GAS (*μ*mol/L)	115.62 ± 12.35	173.21 ± 17.32	16.150	0.001
VIP (*μ*mol/L)	4.27 ± 0.52	8.63 ± 0.96	23.980	0.001
MTL (pg/ml)	295.33 ± 24.53	179.42 ± 17.59	22.740	0.001
CCK (pg/ml)	175.21 ± 15.31	112.73 ± 11.84	18.930	0.001
miR-155	1.53 ± 0.67	0.55 ± 0.51	6.821	0.001
miR-21	1.69 ± 0.72	0.83 ± 0.61	5.357	0.001

**Table 6:** Assignment table.

Factors	Assignment
Alcoholism	Yes = 1, no = 0
GAS (*μ*mol/L)	Data belonged to continuous variables and were analyzed by original data
VIP (*μ*mol/L)	Data belonged to continuous variables and were analyzed by original data
MTL (pg/ml)	Data belonged to continuous variables and were analyzed by original data
CCK (pg/ml)	Data belonged to continuous variables and were analyzed by original data
miR-155	Data belonged to continuous variables and were analyzed by original data
miR-21	Data belonged to continuous variables and were analyzed by original data

**Table 7:** Multivariate logistic regression analysis.

Factors	B	SE	Wals	Sig.	Exp (B)	95% CI of Exp (B)	
						Lower limit	Upper limit
Alcoholism	0.608	0.280	4.709	0.030	3.521	1.061	3.183
GAS (*μ*mol/L)	0.958	0.288	11.056	0.001	5.020	0.218	0.675
VIP (*μ*mol/L)	0.568	0.742	4.996	0.026	3.227	1.072	2.901
MTL (pg/ml)	0.721	0.239	5.705	0.002	4.019	1.467	4.218
CCK (pg/ml)	0.856	0.423	5.512	0.031	4.629	1.353	5.727
miR-155	0.618	0.359	24.14	0.001	6.786	0.824	19.856
miR-21	0.875	0.464	9.473	0.001	2.664	1.347	8.783

## Data Availability

The datasets used and/or analyzed during the current study are available from the corresponding author on reasonable request.
